# Identification of Molecular Regulatory Features and Markers for Acute Type A Aortic Dissection

**DOI:** 10.1155/2021/6697848

**Published:** 2021-04-12

**Authors:** Rui Lian, Guochao Zhang, Shengtao Yan, Lichao Sun, Guoqiang Zhang

**Affiliations:** ^1^Graduate School of Peking Union Medical College, Beijing, China; ^2^Emergency Department, China-Japan Friendship Hospital, Beijing, China; ^3^Department of General Surgery, China-Japan Friendship Hospital, Beijing, China

## Abstract

**Background:**

Acute type A aortic dissection (ATAAD) is one of the most lethal cardiovascular diseases, and its molecular mechanism remains unclear.

**Methods:**

Differentially expressed genes (DEGs) between ATAAD and control were detected by limma R package in GSE52093, GSE153434, GSE98770, and GSE84827, respectively. The coexpression network of DEGs was identified by the WGCNA package. Enrichment analysis was performed for module genes that were positively correlated with ATAAD using clusterProfiler R package. In addition, differentially methylated markers between aortic dissection and control were identified by ChAMP package. After comparing with ATAAD-related genes, a protein-protein interaction (PPI) network was established based on the STRING database. The genes with the highest connectivity were identified as hub genes. Finally, differential immune cell infiltration between ATAAD and control was identified by ssGSEA.

**Results:**

From GSE52093 and GSE153434, 268 module genes were obtained with consistent direction of differential expression and high correlation with ATAAD. They were significantly enriched in T cell activation, HIF-1 signaling pathway, and cell cycle. In addition, 2060 differentially methylated markers were obtained from GSE84827. Among them, 77 methylation markers were ATAAD-related DEGs. Using the PPI network, we identified MYC, ITGA2, RND3, BCL2, and PHLPP2 as hub genes. Finally, we identified significantly differentially infiltrated immune cells in ATAAD.

**Conclusion:**

The hub genes we identified may be regulated by methylation and participate in the development of ATAAD through immune inflammation and oxidative stress response. The findings may provide new insights into the molecular mechanisms and therapeutic targets for ATAAD.

## 1. Introduction

Aortic dissection (AD) is a serious invasive vascular disease with high mortality and limited treatment options [1]. The incidence of aortic dissection ranges from between 3.5 and 6/100,000 person-years in the general population to as high as 10/100,000 person-years in the elderly [2]. Usually, aortic dissection is caused by intimal tear, which further causes blood to flow into the media layer of the aorta, resulting in the separation of the layers within the aortic wall [3]. When the ascending aorta is involved, this dissection is known as Stanford type A aortic dissection (STAAD) [4]. Surgical mortality for acute Stanford type A aortic dissection (ATAAD) is relatively high, despite advances in medical and surgical treatment over the past 30 years [5]. Theoretically, once acute STAAD is diagnosed, patients should undergo emergency surgical treatment immediately [6]. However, limited by geographical, economic, and technical conditions, not all patients can receive timely treatment.

Early clinical symptoms of ATAAD may mimic those of other diseases, such as acute coronary syndrome, pulmonary embolism, or pneumothorax, often leading to delayed diagnosis [7–9]. When ATAAD is detected early and treated promptly, the chance of survival is greatly improved [10–12]. However, even in experienced cardiac centers, the early mortality rate for surgical treatment of acute aortic dissection is around 10%, and many patients still die before surgery [13]. Therefore, we believe that identifying early prognostic biomarkers can leverage patient characteristics and symptoms to optimize treatment strategies [14, 15].

At present, the molecular mechanism of ATAAD remains unclear. Chronic inflammation of the aortic lining has been reported to cause aneurysm growth, leading to aortic dissection [16–18]. In animal models, adventitial inflammation characterized by neutrophil aggregation can promote tissue damage, leading to aortic dilation and rupture [19]. In addition, the medial integrity maintained by collagen and elastin cross-linking is one of the keys in preventing aortic dissection [20]. Bone marrow mesenchymal stem cells are also potential contributors to aortic repair [21].

It is increasingly believed that human disease states are not caused by a single change but by the multifactorial regulation of biological systems [22]. In many cardiovascular diseases, important epigenetic modifications, including methylation, have been shown to affect the development or progression of the disease [23]. Methylation modification of the gene may serve as a diagnostic and prognostic marker in patients with aortic dissection [24].

Weighted gene coexpression network analysis (WGCNA) is a widely used method to build coexpression pairwise correlation matrices [25]. Exclusively based on coexpression analysis, it will better represent genes with a small effect size acting together [26]. WGCNA provides a systems-level insight into the signaling networks that may be associated with a phenotype of interest [27].

The network-based approach provided a powerful option for systematic analysis to identify candidate target genes. The aim of this study was to identify DEGs and related methylation modifications in ATAAD compared with healthy controls. At the same time, the molecular mechanisms involved in gene expression changes were discussed. This study is helpful in identifying new DNA methylation markers and improving both our understanding and the treatment level of ATAAD.

## 2. Materials and Methods

### 2.1. Data Sources

Aortic dissection data were collected from the Gene Expression Omnibus (GEO) database. We screened datasets with a sample size greater than 5. GSE52093 included gene expression data of dissected ascending aorta from patients with acute Stanford type A aortic dissection (*n* = 7) and normal controls (*n* = 5). GSE98770 included gene expression data of dissected ascending aorta from patients with acute type A aortic dissection (ATAAD) (*n* = 6) and gene expression data of nondissected ascending aorta obtained from transplant donors (*n* = 5). GSE153434 included gene expression data of dissected ascending aorta from patients with Stanford type A aortic dissection (*n* = 10) and normal control samples (*n* = 10).

### 2.2. Differential Gene Expression Analysis

The differential expression analysis between aortic dissection and healthy controls was performed by using the R software package limma [28]. The genes with *P* ≤ 0.05 (up-/downregulated) were extracted as differentially expressed genes (DEGs) [29, 30].

### 2.3. WGCNA

A gene coexpression network was constructed through the WGCNA package [31] using differentially expressed genes. The genes with similar expression behavior were divided into different modules. After determining the soft thresholding, the network was developed. Module-trait relationships were calculated using a Pearson correlation between modules and clinical trait. *P* value < 0.05 was regarded as significant.

### 2.4. Enrichment Analysis

Module genes were analyzed using the clusterProfiler R package [32] for Gene Ontology (GO) and Kyoto Encyclopedia of Genes and Genomes (KEGG). The Gene Ontology (GO) enrichment results included the biological process (BP), cellular component (CC), and molecular function (MF) [33]. A term with *P* < 0.05 was considered a functionally enriched term.

### 2.5. Methylation Data Analysis

GSE84274 included methylation profiling of ascending aorta from 6 normal and 12 aortic dissection patients. The difference of methylation sites between aortic dissection and healthy controls was analyzed by the ChAMP software package [34]. Adjust (adj) *P* value < 0.05 was regarded as significant.

### 2.6. PPI Network Construction

We utilized the Search Tool for the Retrieval of Interacting Genes (STRING) database (http://string-db.org) to construct a protein-protein interaction (PPI) network for module genes, with a combined score > 0.4. The PPI network was visualized through Cytoscape software (Version 3.7.0) [35–38]. The genes with the top 5 degrees for connecting other genes in the network were considered as hub genes.

### 2.7. Single-Sample Gene Set Enrichment Analysis (ssGSEA)

To investigate the immune infiltration landscape of acute type A aortic dissection, ssGSEA was performed to evaluate the level of immune infiltration in a sample according to immune cell-specific marker genes [39]. Infiltration levels for immune cells were quantified using the ssGSEA implementation in gsva R package. *P* value < 0.05 was considered significant.

## 3. Results

### 3.1. Coexpression Network of Differentially Expressed Genes

To obtain genes related to acute type A aortic dissection, we compared them with healthy controls. A total of 4913 differentially expressed genes were obtained in GSE52093 (Figure 1(a)). We selected *β* = 18 as the soft thresholding to ensure that the network can obey the scale-free criteria (Figure 1(b)). The created network included three modules (Figure 1(c)). Then, 4682 differentially expressed genes were obtained in GSE153434 (Figure 1(d)). Setting *β* = 10 as the soft thresholding, we got 9 modules (Figures 1(e) and 1(f)).

### 3.2. Biological Functions of Module Genes

The correlation analysis found that MEturquoise (module 2) of GSE52093 had the strongest correlation with ATAAD (Figure 2(a)). MEbrown (module 1), MEyellow (module 5), MEgreen (module 4), and MEblack (module 7) in GSE153434 were positively correlated with ATAAD (Figure 2(b)). Then, we obtained 268 common genes that expressed in the same direction (upregulated or downregulated expression) in these modules (Figure 2(c)). They may have a stronger association with ATAAD. Enrichment analysis revealed that common genes were mainly enriched in response to oxygen levels, T cell activation, leukocyte migration, and NIK/NF-kappaB signaling biological functions (Figure 2(d)). In addition, the p53 signaling pathway, the HIF-1 signaling pathway, the FoxO signaling pathway, and the cell cycle of the KEGG pathways were also significantly enriched (Figure 2(e)).

### 3.3. Methylated ATAAD-Related Genes

By comparing the differences between aortic dissection patients and controls, we obtained 46,845 differentially methylated positions (DMPs) (Figure 3(a)). Most DMPs were concentrated at the chr1 position (Figure 3(b)). We identified 2060 genes with opposite methylation and transcription levels as methylation markers (Figure 3(c)). Interestingly, among these methylation markers, we found that 77 genes were common genes (Figure 3(d)). Using the PPI network, we identified the top five genes with the highest connectivity as hub genes (Figure 4(a)). Compared with the control, MYC, ITGA2, and RND3 were upregulated in ATAAD, and BCL2 and PHLPP2 were downregulated (Figure 4(b)). The AUC values of hub genes were greater than 0.8 in both datasets, which may have a diagnostic role for ATAAD (Figure 4(c)).

### 3.4. Immune Cell Infiltration Difference in ATAAD

Differences in immune cell infiltration were found in ATAAD patients compared with controls (Figure 5(a)). Th1 cells, B cells, T helper cells, T cells, DC, iDC, Tgd, eosinophils, and NK cells were significantly downregulated. The different directions of Th1 cells, Tgd, T cells, T helper cells, iDC, DC, and B cells were consistent in GSE52093, GSE98770, and GSE153434 (Figure 5(b)). These immune cells were clustered into four categories, and there was a positive or negative correlation between the cells (Figure 5(c)). In ATAAD, iDC and macrophages had the strongest positive correlation, while in the control group, iDC and neutrophils had the strongest positive correlation (Figure 5(d)). The correlation analysis results between immune cells and hub genes showed that Th2 cells had the strongest correlation with ITGA2, while NK cells and Th17 cells had the strongest correlation with BCL2 (Figure 5(e)).

## 4. Discussion

Repair of acute type A aortic dissection remains a challenge with high operative mortality [40]. As ATAAD is one of the most elusive and life-threatening vascular diseases, a better understanding of the molecular mechanisms of ATAAD is essential to improve clinical efficacy. In this study, genes with higher correlation with ATAAD were identified by comparing gene expression differences between ATAAD and controls. These genes were mainly associated with immune inflammation. The genes modified by methylation were screened as important genes to construct a PPI network, and five hub genes were identified. In addition, by comparing the difference of immune cell infiltration between ATAAD and control, we also similarly found that immune cells played an important regulatory role in the disease process [41].

Among the ATAAD-related biological functions we identified, T cell activation had been confirmed by other studies [42–44]. Different T cell subsets may play different roles in the development of ATAAD. Elevated white blood cell count is associated with poor prognosis in ATAAD [45, 46]. Inflammatory cells and cytokines, white blood cell count, and neutrophil count have been reported to be responsible for preoperative hypoxemia in ATAAD [47]. Increased inflammatory response is a key factor in promoting the occurrence and development of ATAAD [48]. High inflammatory biomarkers were observed in patients at onset, indicating that the inflammatory response started early in ATAAD [49]. More severe inflammation and oxidative stress reactions occur in obese ATAAD patients [50]. Inflammation and hypoxia are often interdependent [51]. Our findings also suggested that the HIF-1 signaling pathway was activated during ATAAD, thereby aggravating aortic dissection [1]. Therefore, we believe that inflammation and oxidative stress may play an important role in the process of ATAAD.

Notably, upregulated MYC, ITGA2, and RND3 and downregulated BCL2 and PHLPP2 were identified as hub genes of the PPI network. Studies had shown that MYC was indeed upregulated in ATAAD [52]. MYC signaling is involved in vascular smooth muscle cell (VSMC) dysfunction, vasoconstriction, and vascular remodeling in aortic dissection [53]. ITGA2 interacts with collagen in tumors, promotes cell migration, and promotes apoptosis-free resistance [54, 55]. Although there was no direct evidence that ITGA2 was associated with ATAAD, aortic disease was associated with collagen content or structure [56]. It suggested that ITGA2 may act on the development of ATAAD through collagen. In addition, ITGA3 and ITGA5 were identified as new biomarkers for the onset of acute aortic dissection [57]. RND3 played an important role in blocking cell cycle distribution, inhibiting cell growth, and inducing apoptosis and differentiation [58, 59]. Abnormal expression of RND3 may be the main cause of some cardiovascular diseases [60]. The BCL2 protein family influenced the apoptosis of vascular smooth muscle cells in human aortic dissection [61]. PHLPP2 had been reported as a therapeutic target for cancer and cardiovascular diseases [62, 63]. Although no relationship between PHLPP2 and ATAAD had been reported, our findings suggested that its downregulation may be a risk factor for ATAAD.

Most studies used microarray technology to compare diseased and normal aortic tissues and found some signs of ATAAD differentially expressed genes [16, 22]. However, the regulatory mechanisms of differentially expressed genes remain to be determined. The hub genes identified in this study were all modified by methylation. Alterations in gene methylation may mediate the involvement of vascular smooth muscle cells and inflammatory cells in the development of aortic dissection [24]. At present, there are relatively few studies on the regulation of methylation in ATAAD, and we believe that hub genes may be regulated by methylation and thus participate in the progress of ATAAD.

Like other studies, our study also had some limitations. First, these results were obtained only by bioinformatics analysis and were not confirmed by molecular experiments. In addition, although hub genes, potential methylation regulators, and related biological functions of ATAAD had been identified, there was still a long way to go to translate these findings into clinical applications.

It was worth emphasizing that comprehensive network analysis provided a new perspective to understand the molecular basis of ATAAD and promised to elucidate the complex relationship between DEGs in complex diseases. Hub genes were regulated by methylation and participated in the development of ATAAD through immune inflammation and oxidative stress responses. This study will help to identify new DNA methylation markers and improve the understanding and treatment level of ATAAD.

## 5. Conclusion

There were a large number of differentially expressed genes in ATAAD patients, which mainly regulated immune inflammation and oxidative stress functions. In particular, MYC, ITGA2, RND3, BCL2, and PHLPP2 were regulated by methylation in ATAAD. Differential expression of these genes may be associated with the progression of ATAAD, which may be a diagnostic biomarker and a new therapeutic target for ATAAD.

## Figures and Tables

**Figure 1:** WGCNA network for differentially expressed genes. (a) Volcano map of differentially expressed genes between acute type A aortic dissection and controls in GSE52093. Red nodes are significantly upregulated genes, and green nodes are significantly downregulated genes. (b) The soft-threshold power versus scale-free topology model fit index and mean connectivity for GSE52093. The left image shows the scale-free fit index (*y*-axis) as a function of the soft-thresholding power (*x*-axis). The right image shows the average connectivity (degree, *y*-axis) as a function of the soft-thresholding power (*x*-axis). (c) Module clustering tree of differentially expressed genes in GSE52093. (d) Volcano map of differentially expressed genes between acute type A aortic dissection and normal controls in GSE153434. (e) The soft-threshold power versus scale-free topology model fit index and mean connectivity for GSE153434. (f) Module clustering tree of differentially expressed genes in GSE153434.

**Figure 2:** The enrichment analysis of related genes for acute type A aortic dissection. The correlation between module and clinical trait in GSE52093 (a) and in GSE153434 (b). Red represents positive correlation, and blue represents negative correlation. (c) Genes up- or downregulated simultaneously from two datasets in modules which positively correlated with acute type A aortic dissection. (d) The main biological processes of common gene enrichment. (e) The main KEGG pathway of common gene enrichment. Red bars represent upregulated terms, and green bars represent downregulated terms.

**Figure 3:** Acute type A aortic dissection-related methylation markers. (a) Differential methylation positions between aortic dissection patients and controls. (b) Proportion of differentially methylated positions in different chromosomes. (c) Genes whose transcription levels are opposite to the methylation level. (d) Heatmap of the expression of methylation markers in GSE153434. Red nodes are significantly upregulated genes, and blue nodes are significantly downregulated genes.

**Figure 4:** Identification of hub genes for acute type A aortic dissection. (a) The PPI network of 77 methylation markers based on STRING database. (b) The expression of hub genes in GSE153434. (c) The AUC values of hub genes in two datasets. The darker orange color represents a smaller*P*value. The darker red color represents a greater AUC value compared to what the gene has in GSE52093. The darker green color represents a greater AUC value compared to what the gene has in GSE153434.

**Figure 5:** Differences in immune cell infiltration between acute type A aortic dissection and controls. (a) Immune cell infiltration differences between ATAAD and control. Blue columns represent significant differences. Blue lines represent significantly downregulated infiltration of immune cells. (b) Immune cell infiltration differences were validated in three datasets. Red node represents upregulation, and blue node represents downregulation. (c) Cluster diagram of differentially infiltrated immune cells. (d) Correlation of differentially infiltrated immune cells in ATAAD or control. (e) Correlation between differentially infiltrated immune cells and hub genes. Red represents positive correlation between immune cells, and blue line represents negative correlation. ^∗^*P* < 0.05; ^∗∗^*P* < 0.01.

## Data Availability

The data used in our study could be found in GSE52093 and GSE98770.
